The article "Men's Lived Experiences of Breast Cancer and Changes in Occupation" was published in 2023. Journal: Occup Ther Int.

# Men's Lived Experiences of Breast Cancer and Changes in Occupation

**DOI:** 10.1155/2023/9641922

**Published:** 2023-02-13

**Authors:** Ann Marie Potter, Breanne Bentz, Lindsay Crue, Stephanie Leiby, Sogand Bashi, Kaitlin Maguire, Jacob Meyers, Kelsey Mieczkowski

**Affiliations:** ^1^Moravian University, USA; ^2^Elizabethtown College, USA

## Abstract

**Introduction:**

Male breast cancer is rare and frequently diagnosed at later stages of disease with low survival rates. There is a lack of knowledge of how breast cancer impacts men's occupations.

**Objectives:**

This study is aimed at understanding the lived experiences of men with breast cancer and their changes in occupation. *Methodology*. Twenty-four men with breast cancer participated in semistructured phone interviews. Data was open-coded and analyzed for themes. *Findings*. The six major themes are as follows: (1) death as a reality, (2) unique personal insights, (3) social environment, (4) interactions with the healthcare system, (5) decreased engagement in occupations, and (6) finding meaning in new occupations.

**Conclusion:**

The healthcare team can improve the patient experience by discussing and responding to the client's experience throughout the diagnosis, intervention, and survival continuum. The scope of occupational therapy is well suited to address the needs of men with breast cancer to maintain optimal levels of functioning.

## 1. Introduction

Men diagnosed with breast cancer (MBC) face many challenges from diagnosis through the treatment process. This rare disease in men has an approximately 1.2 per 100,000 incidences and 2710 new diagnoses expected in the United States [1, 2]. The median age at diagnosis for MBC is 68 years compared to 62 for women [2]. Despite presenting with similar signs and symptoms as women, male breast cancer often goes unrecognized due to a lack of awareness and male-specific screening protocols [3, 4]. Males tend to be diagnosed at a later age with a more clinically advanced presentation, including larger tumor size, grade, and increased lymph involvement [5–7]. These factors affect the prognosis for males with breast cancer, ultimately creating a lower survival rate when compared to females with the same classification of the disease [3].

A small bank of literature indicates there are a host of emotional and psychosocial challenges faced by men diagnosed with breast cancer [8, 9]. Many men diagnosed with breast cancer reported little knowledge of the disease prior to diagnosis and report a sense of shock when they receive their diagnosis [10–12]. Limited support systems with a high reliance on wives, limited involvement in support groups as they are typically oriented to females, and barriers to accessing health professionals with specialized knowledge of male breast cancer are typical issues reported by MBC [7, 8, 11]. Men are less likely to talk about their diagnosis due to fear of embarrassment related to social acceptability or a perceived threat to their masculinity which may impact coping [9, 10, 13–15]. Stigmatization and marginalization of men with breast cancer has been cited; however recent qualitative studies are not finding this to bare out in the reports of MBC about their experiences with the diagnosis [9, 10, 12]. While the focus of most of the existing literature is on lived experience and coping, Hiltrop et al. [16] examined return to work for MBC. Their qualitative study of fourteen men indicates that men returned to work for a variety of reasons including maintaining normalcy, distraction, socialization, finances, and passion for work.

The article "Men's Lived Experiences of Breast Cancer and Changes in Occupation" was published in 2023. Journal: Occup Ther Int.

Occupational therapists have delved into understanding the female experience of breast cancer and its impact on everyday occupations, occupational engagement, and interaction with the environment [17–19]. These studies highlight the interplay of sequelae related to breast cancer and the effects on the physical abilities to perform activities of daily living and instrumental activities of daily living, role performance, and participation in work and leisure activities. The impact of breast cancer on men's occupations has not been explored. The aim of this research study was to better understand how men experience changes in occupation when diagnosed with breast cancer.

## 2. Materials and Method

### 2.1. Design

This study utilized a qualitative, phenomenological approach to foster the understanding of our male participants' experiences with breast cancer. The use of semistructured interviews allowed researchers to gather personal narratives about the breast cancer experience concerning participation in everyday life while providing participants the opportunity to share personal experiences and perspectives with minimal guidance from the interviewer.

### 2.2. Participants and Recruitment

Recruitment was initiated through the primary author's personal contacts with male breast cancer survivors. We utilized snowball and convenience sampling with assistance from Male Breast Cancer support groups and online organizations. A recruitment flyer was sent to the support organizations and disseminated to members through email blasts. Twenty-nine men responded to the recruitment flyer; twenty-four men completed interviews. The inclusion criteria of this study required that all participants be (1) male; (2) an individual with a personal experience of a breast cancer diagnosis (currently in treatment, in remission, or a survivor); (3) older than 18 years of age; and (4) willing to consent to participate in qualitative interviewing for research-based data collection and use. Participants who could not speak English or communicate verbally were excluded from the study due to the interactional nature of the interviewing process.

The article "Men's Lived Experiences of Breast Cancer and Changes in Occupation" was published in 2023. Journal: Occup Ther Int.

### 2.3. Ethical Considerations

This research study was approved by the Institutional Review Board in January of 2018 as IRBNet ID #1167096-1 at Elizabethtown College, Elizabethtown, PA, USA. All participants completed a verbal informed consent before commencing the interview.

### 2.4. Data Collection

Semistructured telephone interviews were conducted between January and March 2018. A semistructured phone interview format (Table 1) was developed by the research team based on existing literature and theoretical constructs of occupation from the person-environment-occupation model [20]. This approach allowed the researchers to receive relevant and meaningful answers geared to understanding the experience of change in roles and occupation. Before initiating the study's interviews, each team member participated in a pilot interview with a male diagnosed with pancreatic cancer, known to the team. This pilot interview helped researchers understand unforeseen circumstances, such as timing or poor wording of questions, from the perspective of an individual with cancer and helped ensure each interviewer utilized similar styles and probing [21]. The interviews ranged from 10 to 100 minutes.

Research team members, all females, were randomly assigned participants for interviews. Participants in the USA called into a Google Voice number created for this study. International calls used Skype voice. Each interview was recorded, downloaded into a password-protected file, and transcribed using VoiceBase. A research team member checked the transcripts word-for-word with the audio recording and added notes to reflect participants' expressions of emotion. Researchers followed up with participants on multiple occasions to clarify interview responses. Data saturation occurs in collection through a deductive process and inductively during analysis [22]. Data collection saturation occurred when the research team no longer perceived new perspectives shared by participants during the interviews.

### 2.5. Data Analysis

Each transcript was read, open-coded by hand, and themed independently by two members of the primary research team. The primary research team jointly confirmed the themes and conclusions. A second research team of occupational therapy graduate students, 2 female and 1 male, uploaded the cleaned transcripts to Dedoose and performed an additional two rounds of open coding and theming. These results were compared to the first round of coding results and finalized. Inductive thematic saturation [22] was achieved at the point the second research team no longer identified new codes or themes in the data.

The article "Men's Lived Experiences of Breast Cancer and Changes in Occupation" was published in 2023. Journal: Occup Ther Int.

### 2.6. Trustworthiness

The method of researcher triangulation is a validation strategy to view the research data from multiple different points [23]. Multiple researchers conducted interviews to balance the subjective influences of each interviewer throughout the data collection process. Researcher triangulation was also used during data analysis by ensuring that each transcription was individually coded by at least two of the researchers to avoid bias and confirm the consistency of emerging themes and conclusions.

## 3. Results

Twenty-four men completed interviews describing their experience with breast cancer. Five individuals did not follow up with attempted email and telephone communication regarding scheduling and participation.  Table 2 provides an overview of the sample's demographics. Twenty-one participants resided in the United States; the other participants lived in South Africa, Australia, and the Netherlands. The average age of the participants was 57.75 years, the median age was 59 years, and the mode was 70 years of age.

We identified six major themes: (1) death as a reality, (2) unique personal insights, (3) social environment, (4) interactions with the healthcare system, (5) decrease in engagement in occupations, and (6) finding meaning in new occupations.

### 3.1. Death as a Reality

Receiving a potentially life-threatening diagnosis forced ideas of mortality to be consciously considered for many men. This realization of death led to a sense of proactivity that increased their efforts to reach their dreams. Understanding death as a reality positively changed individuals considering their life journey as a gift.

I appreciate life a lot more. Before my cancer, I didn't take life seriously. I took life for granted. I didn't appreciate people in my life and the things I see. So, after cancer, [it] was a good kick in the butt. Just how much you appreciate it, and also made me realize to go after my dreams, chase it, and achieve it. Go after it and every day is a gift. (P-4)

For other men, the reality of receiving a life-threatening diagnosis increased their consciousness of their health, resulting in routine and habit changes.

I think [the diagnosis of cancer] really emphasized that for me the fact that I had vulnerabilities of this nature. That I needed to stay focused a little more on my health in terms of eating properly and losing some weight and getting some more exercise, and that sort of thing. (P-1)

Throughout the experience of being diagnosed with a life-changing disease, all participants experienced an abundance of feelings that forced them to face the challenges ahead. However, these feelings also led to changes in values and beliefs that ultimately shaped them as individuals today.

The article "Men's Lived Experiences of Breast Cancer and Changes in Occupation" was published in 2023. Journal: Occup Ther Int.

### 3.2. Unique Personal Insights

Participants shared personal insights and perceptions and drew on inner strength and external support as their ability to perform roles and occupations was challenged. Support systems provided encouragement and reassurance of the self.

There's a comfort in having your loved ones nearby. That goes beyond having a conversation with them, or having them get coffee for you, or help you clean out the drain [from mastectomy], or whatever. It's the presence that is comforting. (P-1)

Additionally, many men suggested the importance of being open and sharing with support groups. Some men found that by being honest and willing to share their experiences, they could attain the emotional and physical support that they needed.

I found that when I was sharing, it is where the courage and strength came from. When it was uncovered, that I always had in me. I never knew and how important it was for this to come out and to be shared so that people know. (P-19)

I think that being a male and having had breast cancer has given me strength in a way and it's given me purpose because I saw the benefit of speaking out. (P-23)

As treatment progressed, some men reported changes in occupational participation due to side effects, including fatigue, weakness, pain, mood changes, and loss of libido. Feelings of guilt for not being able to complete previous occupations required to maintain a household, perform job responsibilities, or keep the same relationships with family and friends were reported by participants.

I feel very guilty about my ability to do things, you know, with my wife that I used to be able to do more easily (P-15).

Body image was significantly impacted and became a source of stress and fear of what others perceived about their scars, compounding the perception that breast cancer is a women's disease.

I had like prepared this whole Facebook Post, and I feel so stupid saying it now, but I called it chest cancer instead of breast cancer because I was embarrassed. And then my wife convinced me, she's like ‘No, you know, tell it how it is'. So, I had this whole big post ready for Facebook and everything, and I just like held my finger over that post button for five minutes just scared to do it, and my wife grabbed my hand and we did it together… I definitely think it's because society views it as a woman's disease. And I thought people would consider me less of a man because I had breast cancer. (P-21)

In contrast, other men specifically discussed that the mastectomy scars did not affect their ability to engage in social occupations shirtless. One participant described his scar in a positive sense,

The surgery and my scar were going to tell a story. It is my battle wound. The scar is just going to be there, and it's a conversation piece (P-16).

The article "Men's Lived Experiences of Breast Cancer and Changes in Occupation" was published in 2023. Journal: Occup Ther Int.

Personal factors, such as beliefs, values, self-concept, and motivation, were apparent in how participants coped with their initial breast cancer diagnosis and their survivorship journey after that. There were mixed negative and positive self-concepts after receiving a women-dominant breast cancer diagnosis or acquiring a mastectomy scar.

### 3.3. Social Environment

Due to the small population of men with breast cancer experience, many of the participants shared how society has shaped breast cancer into a women's disease. Because of that, they have experienced a sense of stigma behind their unique condition. Many men felt that the public (including healthcare professionals) were unaware and lacked the knowledge to understand breast cancer affecting both men and women.

When I would tell people, that's when it would bother me because they wouldn't believe you. I'd say, “I've got cancer.” “What kind of cancer?” “Breast Cancer.” “Oh, you full of shit, man!”… and I was like, “No, I'm not, you know, I wished I was”… but that is the part that bothers me the most because it happened even at the cancer center where I would get treatment. (P-17)

I told all my friends I had chest cancer, and nobody really questioned what chest cancer is. So, I kind of got away with it there for a couple of years, just calling it chest cancer. And then when I finally came out of the closet, so to speak, and said I had breast cancer, um, people kind of looked at me differently. (P-7)

Social system support came from the family, community, and religious organizations. While help from family and friends was emphasized as necessary throughout these journeys, men expressed the need for more information from the health care team. Due to the rarity of breast cancer in men, many participants lacked communication and support from people in similar situations to their own.

So, I found the men's group. And even though I was the only one with breast cancer, I found it more comfortable and helpful. But I think that fact they had a specific men's group, it was very important in my journey and in my recovery… I really found that women would react to me in a different way (P-23)

All the participants expressed positive feelings towards involvement in the male breast cancer community. Due to shared diagnoses, these men emphasized the importance of connecting with others in similar situations for a network of emotional and information support.

The article "Men's Lived Experiences of Breast Cancer and Changes in Occupation" was published in 2023. Journal: Occup Ther Int.

### 3.4. Interactions with the Healthcare System

The level of awareness and knowledge surrounding male breast cancer can affect men's quality of care from the medical community, ultimately affecting their occupational performance. All the participants acknowledged hindrances and benefits of their interactions with the healthcare system and professionals throughout their journey with breast cancer.

I think the doctor told me one time that I'm at 90 percent success rate where I'm at in treatment, and I said, ‘Well, that's pretty good, and he goes ‘You know, I'll just tell you this is data for women' and I said ‘What about data for me' and he said ‘Well, we don't know. We don't know where you are at.' And I was like, ‘well, that is a bunch of bull,' but that's the way it is because all the concentration is on women. (P-17)

Positive interactions with healthcare providers put the men at ease and built a collaborative relationship.

My oncologist you know he is a wealth of information you ask him a question and his answer is ten minutes long you know can be a short answer of just yes, but he goes on and on and you know everything. You know on the way they kept me at ease and helped me understand everything and made it feel much better. (P-2)

She was now tell me your journey with this with cancer and I was like, oh my god you want to hear what I'm going through. (P-14)

Along with the lack of information for men struggling with breast cancer, participants revealed how the physical environment, printed educational resources, and insurance coverage within the healthcare system are targeted solely toward women. They reported a preponderance of pink, pink ribbons, pink robes, and florally decorated ice packs. The female-oriented healthcare environment negatively impacted the participants. This was not the case for all participants, with some expressing satisfaction with the quality of information and support provided.

I had some issues with my insurance company with getting more tests done. I guess insurance company's computers weren't geared towards men as well, for these kinds of tests, so I got a letter that my sex change was approved, and it kind of destroyed me mentally. (P-14)

The person who had the most impact on my recovery was a onocology nurse navigator, who called me… I had some fairly lengthy conversations about how, you know, patients of her's have reacted to the medications, and to the surgical procedure itself. And provided a level of both knowledge and comfort for me that…and I think a lot of people look at it like no one's ever going through this but me…. So, the recognition that…yes you're…I am unique and my experiences are unique, but there are hundreds of people out there, thousands of people out there, who are going through their own unique path with the same thing. (P-17)

Additional challenges with the healthcare environment centered around the lack of awareness of many healthcare providers, which led to misdiagnosis and delayed diagnosis.

The article "Men's Lived Experiences of Breast Cancer and Changes in Occupation" was published in 2023. Journal: Occup Ther Int.

And the radiologist looked at me, and I can tell that she was kind of nervous. And she starts adjusting the machine, up and down and back and forth. And I could tell she's really nervous, and I can tell she just isn't quite sure what to do with a man. And I actually turned her on I said, ‘you've never done a mammography on a man have you?,' she said ‘No.' I said, ‘OK, why don't you think of me as a flat chested woman.' And do whatever you do for a woman like that. Then it's like a light bulb went on over her head. (P-1)

Overall, the health care environment presented multiple barriers to the men in this study. Several men were fortunate to develop strong connections with their healthcare providers resulting in the sense of trust.

### 3.5. Decrease in Occupational Engagement due to Side Effects

The rigorous treatment protocols for cancer take a toll on the person and the desire to engage in occupations. Side effects of various treatments such as surgery, chemotherapy, radiation, and medication resulted in alterations to daily routines, roles, and participation in occupations.

I used to be able to go to the gym on a Saturday morning and work out and then come home and do yardwork for a few hours, and now I am not capable of that. If I go to the gym Saturday morning, I only have an hour or two left of work in me when I come home. (P-15)

I got behind on housework. Slept a lot. Went from the bed to the couch a lot. I'm not out doing a lot of the things that I used to before (P-2).

I lost interest in my hobbies. I like to fish. I like to play golf. I no longer golf, and I haven't been fishing from the day this started (P-9).

Due to side effects, the inability to work affected many of the men in the study and resulted in disruption and changes to work schedules. Extended periods away from work were frequently required of men who underwent surgery.

When I started having problems with my memory, I kind of lost my confidence in being able to remember because you kind of have followed along like I've asked the customer to do this, and now I'm asking the customer to do that. I didn't want to go back to work, and I didn't go back to work. I never did go back to work. (P-13)

I was off for a couple weeks for my surgery and then when I was going through chemotherapy, I would take off the day of the chemotherapy initially and then towards the end of my chemotherapy um started to catch up with me. So, I was working four days a week when I began my chemotherapy and by the end, I was working three days. (P-15)

Participants reported the impact on their socially ascribed roles of husband and father.

The article "Men's Lived Experiences of Breast Cancer and Changes in Occupation" was published in 2023. Journal: Occup Ther Int.

The aspect of losing my libido was you know that's had an effect on my wife it's denying her an aspect of our marriage, and that's been hard (P-15)

Asking for help was a challenge to masculinity.

Well, I know at work, I've had to get guys to help me do stuff that I never had to have the help to do (P-17)

I'm the breadwinner, you know, I mean my wife works as well, but I'm the main breadwinner, so I need to be out there doing it (P-21).

Overall, the men in our study experienced a decrease in engagement and participation due to the effects of breast cancer and its treatment. Fatigue, memory problems, joint pain, and mobility challenges contributed to altering or completely giving up on activities such as cooking and meal preparation, exercise routines, pet care, auto maintenance, driving, and paid employment. Ultimately, these changes in daily routines, meaningful activities, leisure, work, and roles pushed some of the men to develop new occupations in life.

### 3.6. Finding Meaning in New Occupations

Most participants found meaning in new occupations related to advocacy. This new role centered around building awareness and support for men past, present, and future with breast cancer through public speaking, joining male breast cancer organizations, participating in research, volunteering, and educating others. Some participants expressed the move into advocacy as a natural progression from their profession. Men described themselves in terms of becoming activists. Multiple participants started nonprofit foundations focused on meeting individual and societal needs related to male breast cancer.

The goal was if I can help one male through that, it was done. I achieved my goal. But one person, you know, I mean once you get that satisfaction from that, you just have to keep going. (P-16)

So, part of my support now is trying to educate people and support especially men who have never met another male breast cancer survivor (P-15).

I thought you know what I've left my teaching as an elementary teacher and I'm thinking and realizing my new path is going to be teaching about this. [P-14]

Some expressed finding new occupations through pursuing their dreams. It is not uncommon when being diagnosed with a serious illness such as cancer that a person's life perspective changes. Some men took their diagnosis of breast cancer as an opportunity to engage in occupations that they have always wanted to undertake.

The article "Men's Lived Experiences of Breast Cancer and Changes in Occupation" was published in 2023. Journal: Occup Ther Int.

Each man who participated in our study shared their journey of becoming an advocate for male breast cancer to ensure that men in similar situations had the necessary information and support.

## 4. Discussion

The men in this study revealed the various impacts breast cancer had on their occupations throughout everyday life. They shared what it was like living with a widely female diagnosed disease, the personal implications, and the resulting changes in their occupations. Similarities in cultural norms across the world consisted of different gender norms, including the idea of hegemonic masculinity [24]. This concept divides men and women through stereotypical notions of what it means to be a man, and according to society, breast cancer does not fit into that box. Some men revealed embarrassment and fear of social stigma because they thought they would be perceived as less of a man. This perception is consistent with findings of role strain and stigmatization associated with the “perception of breast cancer as one of being exotic” [8]. Consistent with the work of Rayne et al. [12] and Thompson and Haydock [9] not all participants felt stigma and marginalization and accepted the disease as a diagnosis. Like other recent studies, living with a female's disease left the participants with many unmet health information needs and frequently poorly informed health care providers [5]. These unmet needs prompted participants to assume new roles and occupations in self-advocacy.

Changes in activities of daily living (ADL), instrumental activities of daily living (IADL), social participation, and work were connected to the diagnosis of cancer and side effects including fatigue, pain, physical limitations, support systems, and social perceptions. Declines in functional status, ADLs, and IADLs for all types of cancer survivors, male and female, are well documented [25–28]. ADLs, IADLs, and social participation are domains commonly addressed in oncologic occupational therapy [27, 29]. Current practice trends and evidence support occupational therapy interventions across the cancer continuum to address disease self-management, physical impairments, fatigue, cognition, emotions, energy conservation, work-related issues, and social participation [28–33].

Every participant related a story of their involvement in and the importance of advocacy without a direct question or prompt. This highlights the importance and weight of advocacy in the lives of these men. Self-advocacy is defined as “a means for patients to exert control over complex treatment decisions and uncertain health outcomes, address their unmet needs, and improve their healthcare experience” [34]. In a qualitative study of the self-advocacy experiences of men with cancer, the three major themes managing information, finding the best medical team, and strategic social connections were identified [34]. These themes are consistent with our findings. We viewed concepts of managing information and medical team as separate constructs from advocacy. We interpreted advocacy in the sense of representing a cause and raising awareness. The men in this study viewed the rarity of their diagnosis and the overwhelming focus on female breast cancer the impetus to becoming involved in advocacy with the goal of helping other men to have a better experience and receive better health care. The sense of isolation as a man with cancer, confronting stigma, and seeking others were themes in a study of prostate cancer survivors in Australia [35] and are consistent with the drivers to advocacy expressed in this sample.

The article "Men's Lived Experiences of Breast Cancer and Changes in Occupation" was published in 2023. Journal: Occup Ther Int.

There were high expectations of the men in this study to maintain their employment, causing some men to carry a heavy burden when they had to stop or limit working due to treatment, with participants noting the need to maintain routine and normalcy as well as their professional identity. These themes match those identified in a systematic review of returning to work after breast cancer and other studies including multiple types of cancer [16, 28, 36, 37]. Our results are consistent with the findings of Hiltrop et al. [16], in which male breast cancer survivors in Germany indicated the need to continue with their activities and maintain a sense of normalcy. A study of Italian cancer survivors determined that fatigue, memory issues, and coordinating treatment appointments with work schedule impacted the ability to maintain participation in work activities and are prognostic factors in return to work [36]. Occupational therapists address factors related to return to work with cancer survivors and can fulfill a vital role in promoting and facilitating participation in work [28, 31, 32, 36, 38, 39].

The experience of a decrease in occupational performance led to changes in role fulfillment in these men, such as being a husband, partner, or father. Although the desire to fulfill the expectations of these roles was still present, the demands exceeded their ability to perform these tasks physically. Societal stigmas in the environment pushed the men to challenge concepts of their identity and body image. This effect impacted occupations, as some men reported embarrassment in social occupations with people who were not aware of their diagnosis to avoid further questioning. Social participation is another area frequently addressed by oncology occupational therapists [27, 29, 31, 40].

The article "Men's Lived Experiences of Breast Cancer and Changes in Occupation" was published in 2023. Journal: Occup Ther Int.

The diagnosis of cancer provoked mortal salience, the recognition of the inevitability of death, for these participants. The men reported an abundance of conflicting feelings. The sense of death's imminence prompted many of the participants to reevaluate their lives and make changes in their routines, habits, values, and beliefs. Although cancer is associated with alterations in future expectations, cancer survivors demonstrate resilience and continue to demonstrate positive social well-being and social growth [41].

Trust, communication, and respect are foundations of client- or patient-centered care [42] leading to better health care outcomes. Participants in this study had varied experiences with the healthcare team and environment. Many felt marginalized in environments catering to females, with treatment protocols extrapolated from clinical research and guidelines created for females, and a lack of recognition from their medical providers. Men with breast cancer are frequently viewed as unusual or exotic and report lack of awareness of medical providers which results in limited participation in their own care [8, 10, 11, 14, 24]. Positive support and open communication with medical providers resulted in greater comfort, trust, and comfort in the provider and the treatment process in this study.

Our results concerning the ability to fulfill required and desired roles were consistent with findings from a previous qualitative study of women with breast cancer and men with bowel cancer highlighting the importance of social, emotional, and physical support in maintaining a sense of self-worth [17–19, 30]. Finding meaning in engagement in new occupations was a common theme in both genders dealing with breast cancer. New occupations allow those living with breast cancer to replace occupations that were once meaningful but can no longer be performed nor desired. The experience of a life-threatening condition can compromise an individual's identity, engagement in social relationships, and ability to fulfill roles of everyday life. Engagement in modified or new occupations may be a coping response to the psychological challenges presented by cancer [43].

### 4.1. Strengths and Limitations

The robust sample size of 24 provided a significant amount of data for a comprehensive understanding of the lived experience of the participants. This study is the first of its kind to examine the occupations of men with breast cancer. Triangulation through the data collection and analysis process decreases bias and increases trustworthiness.

The article "Men's Lived Experiences of Breast Cancer and Changes in Occupation" was published in 2023. Journal: Occup Ther Int.

Convenience sampling through support groups is a significant limitation of this study. Men involved in the support groups were not fully representative of the entire population of male breast cancer. Bias in the results is evident in the fact that every participant in this study was involved in advocacy and support groups. The study does not reflect the experiences of men not involved in advocacy and support related to a breast cancer diagnosis. Participants discussed their path to advocacy involvement and data does not provide insight into why some men do not go into advocacy and support groups. Self-selection limits generalizability of the study.

Participants in this study were at various stages of the cancer survivor trajectory. This study does not reflect the different experiences associated with different stages of the breast cancer treatment and survivorship timeline. Additional research is needed to explore the specific relationship between disease sequelae and occupational performance, changes in occupational performance overtime for cancers survivors, and the efficacy of occupational therapy to address changes.

## 5. Conclusion

The aim of this research study was to better understand how men experience changes in occupation when diagnosed with breast cancer. The lived experiences shared by the men in this study provide insight into the physical, emotional, and social challenges they faced from diagnosis through treatment and into the survival phase. Participation in meaningful occupations were altered for all participants by the experience of male breast cancer. Participants discussed ways of adapting, such as seeking out needed support in their environment or engaging in new occupations such as becoming involved in advocacy groups. Evidence from this study supports that a sense of self, identity, and ability to interact with the social environment strengthened engagement in meaningful occupations. The lived experiences of the men in our study were like the lived experiences of women with breast cancer, men with prostate cancer, and bowel cancer survivors [17, 18, 30, 35]. Stigma related to having a diagnosis of a disease associated with women created challenges in diagnosis, medical treatment, and in social environments.

All health care providers must maintain a client-centered approach that provides space for the unique experiences of each client and not fall into stereotyping which may stigmatize or marginalize the client. Occupational therapy has the ability promote engagement in meaningful occupations and therefore promote overall health and well-being [27, 29, 33, 39] in the lives of men affected by breast cancer through understanding the unique barriers and successes men in this study described. The men in this study expressed instances where they did not feel welcome in the healthcare environment and their health care providers were not well versed in treatment of male breast cancer. Only through a client-centered and occupation-based approach will occupational therapy benefit clients to achieve optimal occupational engagement [20].

The article "Men's Lived Experiences of Breast Cancer and Changes in Occupation" was published in 2023. Journal: Occup Ther Int.

## Figures and Tables

**Table 1:** Interview guide.

(1) Tell me about your experience with breast cancer from the time you were diagnosed until now. (Probes: Diagnosis/Symptoms, Treatment, Recovery)
(2) Talk about the first thoughts that went through your mind when your doctor confirmed you had breast cancer. (Probe: How did the diagnosis of breast cancer change the way you saw yourself?)
(3) What aspects of your life have changed since you have had breast cancer? (Probes: What aspects of your everyday life changed? What specific changes have you noticed in your ability to complete the duties of your everyday life as a result of your diagnosis of breast cancer? Why were these tasks difficult? To what symptoms do you attribute these changes? Roles, Routines, Leisure, Work)
(4) How has your sense of self changed through your experiences of breast cancer? (Probe: How did this experience change your values or beliefs?)
(5) Explain how your support system has looked throughout your journey with breast cancer?
(6) Tell me about your treatment team and the healthcare professionals that you came into contact with when receiving treatments? (Probe: Which ones had the most impact toward your recovery?)
(7) Have you had periods of time in which you felt differently within social or family situations? (Yes/No) (Probes: Please describe a specific time or situation in which you felt this way. Please describe specific thoughts and feelings during this time. How would you handle it if you felt like this?)

**Table 2:** Demographics.

	*N* = 24	(%)
*Age (years)*		
<50	7	29.2
50-65	9	37.5
>65	8	33.3
*Years since diagnosis*		
≤5	10	41.7
6-14	12	50.0
≥15	2	8.3
*Stage of breast cancer*		
Stage I	6	25.0
Stage II	10	41.7
Stage III	4	16.7
Stage IV	3	12.5
Not specified	1	4.1
*Undergoing treatment during study*		
Yes	12	50.0
No/completed treatment	12	50.0
*Employment status at time of treatment*		
Employed full-time^∗^	15	62.6
Retired	7	29.1
Not employed	2	8.3
*Relationship status*		
Single	2	8.3
In relationship	21	87.5
Widowed	1	4.1
*Ethnicity*		
White	22	91.8
Hispanic	1	4.1
Not specified	1	4.1

^∗^Some participants indicated taking a leave of absence or decreasing work hours while undergoing treatment.

The article "Men's Lived Experiences of Breast Cancer and Changes in Occupation" was published in 2023. Journal: Occup Ther Int.

## Data Availability

Data are available through a request to the corresponding author Ann Marie Potter pottera@moravian.edu.
